The article "The Construction of a Diversified and Open Teacher Education System Management System That Integrates Public Mental Health" was retracted in 2023. Reasons: signs of a paper mill; suspected computer-generated content; unreliable results or conclusions; concerns about the data.

# The Construction of a Diversified and Open Teacher Education System Management System That Integrates Public Mental Health

**DOI:** 10.1155/2022/9269412

**Published:** 2022-08-17

**Authors:** Jixin Qin

**Affiliations:** School of Information Science and Technology, Nantong University, Nantong, Jiangsu 226019, China

## Abstract

The teacher education management system is crucial to the operation of the teacher education system (TES). It is the core institutional system of the TES, which stipulates the management authority and functional scope of the relevant departments of the TES. After the new pluralistic and open TES is formed, the original management system must be adjusted accordingly. In this context, this article integrates public mental health (PMH) into the diversified and open management system of TES and then uses a neural network to evaluate and complete the following tasks: (1) this article introduces the development status of diversified and open TES management systems at home and abroad and the importance of public psychology courses to teacher education. (2) The framework of TES integrating PMH is proposed, and then the principles of BPNN and gray wolf optimization (GWO) algorithm are introduced, and the IGWO-BPNN model is constructed accordingly. (3) The convergence and fitness of the IGWO-BP model and the GWO-BP model are compared through experiments, which proves the superiority of the performance of the IGWO-BP model. The optimal model is constructed by selecting parameters, and then the output of the model is compared with the expert evaluation results, and the error is small. It is proved that the model has superior performance in evaluating the professional quality of teacher education. (4) This article selects three professional quality evaluation indicators of teacher education to compare the changes before and after the integration of PMH. The results show that the proposed diversified and open management system of TES integrating PMH can effectively improve the professional quality of teachers in all aspects.

## 1. Introduction

Teacher education, as a professional education for cultivating teachers, has gone through more than 100 years of ups and downs in my country and has formed a TES with independent normal colleges as the main body [1]. Undoubtedly, the relatively independent TES has sent a large number of teachers to schools at all levels, especially primary and secondary schools, and has made significant contributions to stabilizing the teaching force and supporting the development of basic education. However, this directional teacher training model of directional enrollment, directional training, and directional distribution also brings about the closed nature of teacher education and the singleness of teacher sources, which affects the improvement of the quality of the teaching staff [2, 3]. Obviously, it cannot fully adapt to the new situation, especially the need for high-quality talents in the era of the knowledge economy, and the TES is in a rigid predicament. The only option to get out of the predicament is to change from a directional training model to a diversified and open TES. This is also the trend of teacher education development in major developed countries in the world [4–6]. In order to overcome the shortcomings of the closed teacher education system and improve the quality of teacher training, the United States took the lead in reforming the closed TES as early as the 1940s and implemented an open TES. Subsequently, many countries followed the example of the United States and successively reformed the closed higher normal education system and implemented a diverse and open TSE that includes comprehensive universities or nonnormal colleges, normal colleges, and education colleges participating in the training of primary and secondary school teachers [7, 8]. Judging from decades of development practice, a diverse and open TES does play an important role in improving the quality of teacher education and is also conducive to improving people's self-ability, reflecting the idea that education should focus on people's development [9]. My country's higher education began to reform its management system in accordance with the policy of “co-construction, adjustment, cooperation and merger” since 1992. After a new round of mergers and adjustments of colleges and universities, we can see that a diversified and open TES has gradually formed in which comprehensive universities participate in the training of primary and secondary school teachers. That is to say, after a new round of adjustment and reform of the management system of colleges and universities, as well as the policy encouragement of the two “decisions,” the current and future teacher education in our country is forming an independent set of various normal colleges and universities. It is an open TES that trains primary and secondary school teachers in a multichannel, multistandard, and multiform manner with the participation of the main body and other educational institutions [10–12]. This system consists of four parts: first, higher normal colleges and universities set up independently; second, comprehensive and other nonnormal higher education institutions participating in the education and training of middle school teachers; third, normal colleges and universities are gradually divided into comprehensive and other types of higher education institutions; fourth, normal colleges and universities that are merged into comprehensive institutions of higher learning or nonnormal institutions of higher learning and continue to train middle school teachers. Judging from the history of teacher education and the characteristics of the development of teacher education in the world, the trend of my country's TES is bound to change from directional closed teacher education to a nondirectional open and diversified TES [13–15]. The management system of higher education refers to the leadership division of labor, institutional setup, affiliation, management authority, and management content within the higher education system, as well as the composition status and function of various systems, laws, and regulations that are compatible with it [16]. The original management system of higher normal education in our country is a two-level management system at the central and provincial levels. At the central level, the Department of Teacher Education of the Ministry of Education, on behalf of the central government, implements leadership management over the relevant management institutions of the subordinate normal colleges and local education administrative departments. The Higher Education Office of the local education administrative department shall, on behalf of the local government, exercise leadership over the normal colleges and universities affiliated with the province. This management system is accompanied by an independent closed TES and is adapted to the directional and closed TES in the past. It played an important role in the development of teacher education at that time and even the development of the whole education [17]. However, with the transformation of my country's TES from a closed type to an open type, after the formation of the new pluralistic and open TES, this management system is obviously not suitable for the new TES. It is necessary to adjust or rebuild a new management system to ensure the healthy, orderly, and high-quality development of teacher education [18]. In this context, this article integrates public mental health into the diversified and open management system of TES, constructs the evaluation index of teacher education ability, and then uses a neural network to evaluate and to prove the effectiveness of the management system of this TES.

## 2. Related Work

It is not only an inevitable trend but also a process of gradual realization that my country's teacher education model is moving toward a high-level, diversified and open goal. The new teacher education policy clarifies the future development direction of my country's teacher education. However, after years of practice, the reality is not satisfactory [19]. Reference [20] proposed that to seriously reflect on the experience and problems of the transition from teacher education to teacher education in my country, we must consider the reality of China's vast territory and great regional development differences and build a comprehensive and open teacher education model. Implementing open teacher education is not about weakening or abolishing normal colleges. Our task is to actively reform, improve, and build a modern TES with Chinese characteristics that meet the needs of education reform and improve the quality of teacher training [21]. Reference [22] believed that open teacher education should take the development path of “one main and multiple” in which teachers' education is run by comprehensive universities and professional colleges. The task of teacher training and continuing education is quite heavy. Teacher colleges undertake a major mission and need to further play the main role of normal colleges in teacher education. For example, according to [23], it is not apparent what our nation's transformation of teacher education is for and there is not enough evidence to back it up. This contradicts the need to improve the quality of teachers in our country. Normal colleges and universities should also take over as the primary source of teacher training over the long term, and the autonomous system of teacher education must be maintained for as long as possible while simultaneously implementing openness in teacher training. There are two main forms of open teacher education institutions: one is to use the original higher normal schools as the main body to expand their professional fields or to adjust and merge institutions to develop into comprehensive institutions. Second, professional colleges such as comprehensive universities, art colleges, sports colleges, and ethnic colleges participate in teacher education [24]. As the main body of teacher education, normal colleges and universities should develop from a single type to a comprehensive type and form a modular teacher education specialization model. The modular teacher education specialization model refers to the development from a single type to a comprehensive type under the conditions of the existing teacher education. By adjusting the curriculum structure, the curriculum is divided into several modules to increase the teaching content and time of educational science literacy education, to realize the discipline specialization and education specialization of teacher reserve talents [25]. Teacher education also has some special tasks, which is to train teachers of comprehensive junior high school courses, teachers of science courses, primary school teachers, kindergarten teachers, and teachers of special children. These special circumstances should be considered when designing curriculum modules. The mode of cultivation can be varied. However, it is necessary to formulate teacher training programs and teacher education curriculum standards of different specifications. The four major modules of general education, subject education, teacher professional education, and internship are indispensable [26]. Reference [27] proposed that the original normal colleges can be merged with other professional colleges to form a new comprehensive university. This can bring good opportunities to the development of teacher education. It can rely on the multidisciplinary and high-level academic advantages of comprehensive universities to make teacher education from closed to open and to provide knowledge, academics, and information for training high-level teachers and other foundations and conditions. As comprehensive universities and professional colleges that participate in teacher education in a diversified manner, teacher education can take the path of staged teacher professional training. Teachers' subject specialization and education specialization are carried out in stages, which can better achieve the goal of teacher specialization and is a feasible idea to promote the diversification of teacher education. The new management system of teacher education should be in line with the socialist market economic system and political system reform, in line with the law of education's own development and the development trend of international higher education reform [28, 29]. References [30, 31] believed that the management system of teacher education implements the central and local secondary centralized management system at the macro level. The Division of Teacher Education is mainly responsible for managing specific business, principles, and policies, conducting macrocontrol and policy adjustment on the development scale of teacher education and improving the quality of training, strengthening the construction of educational science disciplines, and summarizing and exchanging the training experience of teacher education in various universities. Experts supervise, inspect, guide, and evaluate the quality of teacher education; review and approve the conditions and qualifications of higher education institutions directly under the Ministry of Education to participate in the education and training of primary and secondary school teachers; take charge of leading the granting and inspection of teacher qualifications across the country. The local area is under the overall management of the Department of Education, and the specific business is under the responsibility of the Higher Education Teacher Education Office. It accepts the guidance of the Teacher Training Department of the Ministry of Education in terms of business. It is mainly responsible for the development planning of teacher education in the region and guides the teacher education and training work and quality inspection work in colleges.

## 3. Method

### 3.1. TES Frame Integrating Public Mental Health

Psychology is a core course in the teacher education professional curriculum system and plays an important role in the training of teachers. The “Opinions of the Ministry of Education on Vigorously Promoting the Reform of Teacher Education Curriculum” promulgated in 2011 emphasized that training high-quality professional teachers needs to strengthen the practice link, focus on the training of teachers' educational and teaching ability, and improve teachers' practical ability. Therefore, improving the practicality of psychology teaching is an important part of achieving the goal of high-quality teacher training. The so-called practical teaching often refers to practical activities in military training, practice, social practice, and graduation thesis. This definition easily leads to the misunderstanding that practical teaching activities and classroom teaching activities operate independently and are separated from each other. However, even the relatively theoretical aspects of learning, such as psychological concepts, knowledge, and principles, are not isolated from practice. For scientific research, there is no theory that is not related to practice, only practice that does not reach the level of theoretical abstraction. Psychology, as a research object, comes from a science of practice, and it is inextricably linked with the subject and object of practice, that is, people or learners. Therefore, the practical forms of psychology teaching should be richer and more diverse, not just limited to common educational observation, educational practice, and social practice. There are three types of teaching practice divided. Whether it is the cognitive practice of individual dialogue with the objective world, the social practice of dialogue with others, or the moral and emotional practice of dialogue with oneself, we believe that all practical teaching activities belong to the category of practical teaching. Therefore, in the teaching process, teachers make psychological science problems live, contextualize, and socialize and let students participate in various interactions, or teachers lead students to laboratories, primary and secondary schools, and enter the vast world of society, allowing students to do it by themselves. Operation, observation, solving practical problems, participating in social practice, and doing scientific research can all be regarded as practical teaching of psychology. For a long time, students have generally reported that psychology courses have many professional terms, abstract theory, and the existence of complex curriculum content systems. At present, the total class hours of public psychology for teacher education majors in most colleges and universities in China are usually only 56–64 classes. In a limited time, teachers have a heavy teaching task. Moreover, it is often necessary to teach in large classes with fifty to sixty people or even hundreds of people. It is difficult to organize large-scale and regular educational internships and social practice activities during the teaching period. Most of the teaching methods are based on traditional teaching methods. If teachers do not pay enough attention to the practicality of classroom teaching, and the teaching still focuses on theoretical exposition and lacks interest, it will obviously further alienate the relationship between the curriculum and the learners. The teaching effect is more difficult to meet the expectations of students. In recent years, many beneficial reforms and practices have been carried out in China in terms of curriculum content system and teaching methods, trying to improve the practicality of public psychology teaching content and teaching process. An extensive collection of newly developed teaching materials has been assembled together with a number of innovative new techniques of instruction such as seminar methods, problem-based learning, and multimedia-based learning. These measures have eased the contradiction between psychology teaching and learning to a certain extent. However, under the current situation that the Ministry of Education has repeatedly emphasized practical teaching, required to increase the proportion of practical teaching and strengthen the work of practical education in colleges, the teaching reform idea of distinguishing different types of practical education advocated by the Ministry of Education has not received enough attention. In the teaching of psychology courses, we make full use of various teaching methods such as simulated classrooms, on-site teaching, situational teaching, and case analysis. It is a problem worthy of further study to enhance the learning interest of normal students and improve the teaching efficiency to demonstrate the practicality, intuition, image, and interest of public psychology classroom teaching. Based on the diverse viewpoints of the practice teaching form of public psychology, this article constructs a framework of TES that integrates PMH, as shown in Figure 1.

### 3.2. BP Neural Network

Based on error backpropagation and self-adjustment, BPNN is a feedforward network with several layers that can learn and adapt to new situations. As one of the most extensively used neural network models, it has a lot of support. The BPNN can not only perform self-learning and form a large number of input and output mapping relationships but also use its unique “black box” to perform nonlinear fitting on multiple sets of training data to find out the laws between the data, without giving prior mapping relationship between data. BPNN is a feedforward neural network with many layers. The signal travels forward, while the mistake travels backward as a result of this phenomenon. It is now the most used neural network. The structure of the BPNN model is commonly separated into three components, namely, input, hidden, and output layers. In order to employ the backpropagation of error corrections to continually modify the network weights and thresholds in order to reduce the error, it trains the samples. It is possible to slip into local minima, sluggish convergence, and “overfitting” using BPNN, despite its simple structure and excellent nonlinear fitting capacity.  Figure 2 is the basic structure of the BP neural network.

If *j* basic neurons are given, it can mainly achieve three basic and most important functions: weighting, summation, and transfer. *X*=[*x*_1_, *x*_2_,…, *x*_*n*_] represents the input from neurons 1,2,…*i*,…, *n* respectively; *W*=[*w*_*j*1_, *w*_*j*2_,…*w*_*ji*_,…, *w*_*jn*_] is the weight; *b*_*j*_ is the threshold; *f* is the transfer function; *y*_*j*_ is the output of the jth neuron. The net input value *S* of the jth neuron is

(1) $$\begin{array}{c} S_{j}=\sum_{i=1}^{n}w_{ji}x_{i}=W_{j}X. \end{array}$$

*S*_*j*_ can get *y*_*j*_ through the transfer function *f*:

(2) $$\begin{array}{c} y_{j}=f\left(S_{j}\right)=f\left(\sum_{i=0}^{n}w_{ji}x_{i}\right)=F\left(W_{j}X\right), \end{array}$$

where *f* is a bounded monotone increasing function.

The information exchange between neurons in BPNN relies entirely on the transfer function, and the commonly used transfer functions are as follows. There are no restrictions on what you may put into the Log-Sigmoid function; it returns the range [0, 1]. Tansig is similar to the Log-Sigmoid function in that it accepts any input value and returns a value between −1 and 1. The inputs and outputs of Purelin may be whatever you want them to be. Hidden layers in the BPNN are possible. Any value may be generated by a complete neural network if the hidden layer and output layer both use sigmoid transfer functions.

Forward data propagation and backward error signal propagation make up the BP algorithm. Each layer's neurons only communicate with those in the below layer in the forward propagation direction: input layer, hidden layer, and output layer. If the result cannot output the target value, the calculation error realizes the reverse feedback. When the two processes are repeatedly crossed, the weight vector is constantly adjusted in the space, and the error function also implements the gradient descent strategy, and iterative operations are continuously performed to minimize the network error. The following are two ways for BPNN to propagate:

(1) Forward propagation: it is assumed that the input layer of the BPNN has *n* nodes, the hidden layer has *q* nodes, and the output layer has *m* nodes. The weight between the input layer and the hidden layer is *v*_*ki*_, and the weight between the hidden layer and the output layer is *w*_*jk*_. The transfer function of the hidden layer is *f*_1_, and the transfer function of the output layer is *f*_2_, then the output of the hidden layer node is as follows:
  (3) $$\begin{array}{c} Z_{k}=f_{1}\left(\sum_{i=0}^{n}v_{ki}x_{i}\right),\;k=1,2,\ldots ,q. \end{array}$$
The output of the output layer is as follows:
  (4) $$\begin{array}{c} y_{j}=f_{2}\left(\sum_{k=0}^{q}w_{jk}z_{i}\right),\;j=1,2,\ldots ,m. \end{array}$$
So far, the BPNN has completed the mapping of the n-dimensional space vector to the m-dimensional space.
(2) Backpropagation: input *p* learning samples, and the output *y*_*j*_^*γ*^ is obtained after the pth sample is input into the network. Using the squared error function, the pth sample error can be obtained:
  (5) $$\begin{array}{c} E_{\gamma }=\frac{1}{2}{\left(\sum_{j=1}^{m}t_{j}^{\gamma }-y_{j}^{\gamma }\right)}^{2}, \end{array}$$
where *t*_*j*_^*γ*^ is the expected output.
For *p* samples, the global error is as follows:
  (6) $$\begin{array}{c} E=\frac{1}{2}\sum_{\gamma }^{p}\sum_{j=1}^{m}{\left(t_{j}^{\gamma }-y_{j}^{\gamma }\right)}^{2}=\sum_{\gamma }^{p}E_{\gamma }. \end{array}$$
The weights of the output layer use the cumulative error BP algorithm to adjust *w*_*jk*_ to make the global error *E* smaller:
  (7) $$\begin{array}{c} \Delta w_{jk}=-\eta \frac{\partial E}{\partial w_{jk}}=-\eta \frac{1}{2}\frac{\partial }{\partial w_{jk}}\left(\sum_{\gamma }^{p}E_{\gamma }\right)=\sum_{\gamma =1}^{p}\left(-\eta \frac{\partial E_{\gamma }}{\partial w_{jk}}\right), \end{array}$$
where *η* is the learning rate.

(8) $$\begin{array}{c} \delta_{yj}=-\frac{\partial E_{\gamma }}{\partial S_{j}}=-\frac{\partial E_{\gamma }}{\partial y_{j}}\cdot \frac{\partial y_{j}}{\partial S_{j}}, \end{array}$$

where *δ*_*yj*_ is the error signal. So the output layer weight adjustment formula is as follows:

(9) $$\begin{array}{c} \Delta w_{jk}=\sum_{\gamma =1}^{p}\sum_{j=1}^{m}\eta \left(t_{j}^{\gamma }-y_{j}^{\gamma }\right)f_{2}^{\prime }\left(S_{j}\right)z_{k}, \end{array}$$

where Δ*w*_*jk*_ is the variation of the output layer weights.

Changes in hidden layer weights are as follows:

(10) $$\begin{array}{c} \Delta v_{ki}=-\eta \frac{\partial E}{\partial v_{ki}}=-\eta \frac{\partial }{\partial v_{ki}}\left(\sum_{\gamma =1}^{p}E_{\gamma }\right)=\sum_{\gamma =1}^{p}\left(-\eta \frac{\partial E_{\gamma }}{\partial v_{ki}}\right), \end{array}$$

where Δ*v*_*ki*_ is the variation of the hidden layer weights.

(11) $$\begin{array}{c} \delta_{zj}=-\frac{\partial E_{\gamma }}{\partial S_{k}}=-\frac{\partial E_{\gamma }}{\partial z_{k}}\cdot \frac{\partial z_{k}}{\partial S_{k}}, \end{array}$$

where *δ*_*zj*_ is the error signal. Thus, the hidden layer weight adjustment formula is obtained as follows:

(12) $$\begin{array}{c} \Delta v_{ki}=\sum_{\gamma =1}^{p}\sum_{j=1}^{m}\eta \left(t_{j}^{\gamma }-y_{j}^{\gamma }\right)f_{2}^{\prime }\left(S_{j}\right)\Delta v_{ki}f_{1}^{\prime }\left(S_{k}\right)\cdot x_{i}, \end{array}$$

where Δ*v*_*ki*_ is the variation of the hidden layer weights.

The emergence of the BPNN algorithm is to solve the situation of linear inseparability. It uses the principle of backpropagation of errors, changes the traditional network structure, introduces new layers and logic, and basically solves the nonlinear classification problem. With the BPNN algorithm, learning takes place in two stages: forward propagation of the signal and reverse propagation of the mistake. Passed from the input layer to the hidden layer, and then communicated to the output layer, are input samples. It is possible that the output error will be disseminated to the neurons in each layer, which will then utilize the error signal to alter the weights and continually adjust as a result of propagating it via the hidden layer. Only repeat forward propagation and error backpropagation if there is a tiny mistake or the predetermined iteration duration and a number of iterations have been met.

### 3.3. Intelligent Optimization Algorithm

#### 3.3.1. Gray Wolf Optimization Algorithm

The gray wolf optimization (GWO) algorithm is a swarm intelligence optimization algorithm that simulates gray wolves to hunt their prey. Whether a gray wolf is swimming or running, the closer a wolf is to its prey, the easier it is for the wolf to capture the prey, that is, the greater the fitness of the wolf. During the operation, the calculated fitness values of gray wolves will be sorted, and four types of gray wolves will be divided according to the fitness values from large to small: the optimal gray wolf *α* (head wolf), the second-best gray wolf *β* and the third best gray wolf is *σ*, and the last gray wolf is *w*. These four kinds of gray wolves represent different social classes in the wolf pack, corresponding to the leader *α*, the deputy leader *β*, the small leader *σ*, and the common gray wolf *w* in the population, respectively. In the process of optimization, the position of the optimal gray wolf *α* represents the optimal solution, and all the gray wolves constantly roam and move toward the position of the optimal solution. With the iteration of the algebra, the position of the wolf pack is continuously updated, and finally, the position of the prey is reached, and the position of the prey is the optimal solution. The optimization principle of the algorithm is as follows: in the entire population, the population number is N, the number of weight thresholds to be optimized is dim, and the objective function is the prey concentration value perceived by the gray wolf, that is, the fitness. The optimal gray wolf *α* is the gray wolf with the greatest fitness, but it is not specific. The position of each gray wolf will be updated during the marching project, and when a gray wolf with greater fitness appears, the head wolf will be replaced. In addition, the gray wolf *β* and the gray wolf *σ*, and the remaining gray wolf is *w*, will also be updated according to the change in fitness value. In the D-dimensional search space of the gray wolf population, we set the position of the ith wolf in the gray wolf population as *X*, where  *i* ∈ (1,  2,  3,…, *N*). The following is a description of the behavior of the gray wolf narrowing the search area, constantly approaching its prey, and taking a siege. Calculate the position of the prey and the distance vector *D* between the individual gray wolf and the prey:

(13) $$\begin{array}{c} D=|C\cdot X_{p}\left(t\right)-X\left(t\right)|\;C=2r_{1}, \end{array}$$

where *X*_*p*_(*t*) is the position of the t-th generation of prey; *X*(*t*) is the position of the t-th generation of gray wolves; *C* is the vector coefficient; *r*_1_ is a random number of [0, 1].

#### 3.3.2. Improved Gray Wolf Optimization Algorithm

In the GWO algorithm, the original iteration coefficient *a* will decrease linearly until it is 0 in the iterative process, but in the actual optimization process, the gray wolf algorithm does not converge linearly, so the original iteration coefficient *a* cannot better represent the algorithm's optimization process. To this end, this article uses an improved nonlinear convergence method.

(1) Iteration coefficient *a*:

(14) $$\begin{array}{c} a=2-2\left(\frac{1}{e-1}\times \left(\frac{l}{e^{\text{Max}Iter}}-1\right)\right), \end{array}$$

where *e* is a natural constant, *l* is the current number of iterations, and Max*Iter* is the maximum number of iterations.

In the optimization process of the gray wolf algorithm, the *α* wolf is not necessarily the global optimal point, and with the continuous iteration of the wolf group, the algorithm is likely to fall into the local optimal. In this article, the proportional weight *W* is introduced to strengthen the global search ability of the algorithm.

(2) Introduce the weight W. The formula for calculating the proportional weight is as follows:

(15) $$\begin{array}{c} W_{1}=\frac{|X_{1}|}{|X_{1}|+|X_{2}|+|X_{3}|}. \end{array}$$

### 3.4. Improved Gray Wolf Optimized Algorithm Combined with BPNN Model

This article will use the improved gray wolf algorithm optimization (IGWO) combined with BPNN to establish the prediction model of IGWO-BP. The idea is to optimize the weight and threshold of the BPNN and assign the optimal weight threshold to the BPNN to complete the evaluation. Among them, the weights and thresholds of the BPNN represent the location information of the gray wolves. Through a series of behaviors such as the walking and hunting of the gray wolves, the entire wolves continuously update their position, and finally, the optimal weight threshold required by the BPNN can be obtained. The steps of the IGWO-BP neural network are as follows:

1. Determining the neural network structure: the main purpose is to determine the number of hidden layers, and the BPNN model with a single hidden layer can approximate any nonlinear mapping relationship, so this article adopts a three-layer network.
2. Gray wolf population initialization: the individual dimension dim of gray wolves is determined by the number of weight thresholds to be optimized, the population size N, and the maximum number of iterations, the upper and lower bounds of the search space of gray wolves are determined, and the location information of wolves is randomly generated.
3. Determine the transfer function, training function, and fitness function of the neural network. The network transfer function is a tansig function, the network training function is trainlm, and the fitness function is the mean square error (MSE) between the predicted output and the actual value.
4. Calculate the fitness and sort the fitness value. And classify the gray wolf group: the best gray wolf *α*, the gray wolf *β*, the gray wolf *σ*, the gray wolf *w*, and update the positions and parameters of all gray wolves.
5. Obtain and record the error between the training sample and the test sample and the position of the corresponding optimal gray wolf *α*.
6. Determine whether the set error is met or the maximum number of iterations is reached; otherwise, steps 4 to 6 will be repeated until the conditions are met.
7. The returned result is the optimal gray wolf *α* position and the corresponding minimum error.

### 3.5. Teacher Education Evaluation Index Integrating Public Mental Health

The construction of the evaluation index system for the professional quality of education teachers is a systematic project, and it is a process of specifying the evaluation attributes based on the decomposition of evaluation objectives layer by layer. This process includes determining the evaluation object, determining the evaluation target, and preliminarily drawing up the evaluation index system

1. Determining the evaluation object: first, the evaluation object of the evaluation index system must be clearly defined. The professional quality of vocational education instructors is the assessment item for the index system used to assess education teachers' professional quality. Therefore, the evaluation index system must be able to reflect the generality and particularity of the professional quality of vocational education teachers.
2. Determining the evaluation objectives: for vocational education instructors, the assessment objectives of professional quality should be aligned with educational and personnel training goals of the nation and schools, and the teaching and professional development goals of vocational teachers. The evaluation may only be used to help improve the professional quality of vocational education instructors if it is done in accordance with these aims.
3. Preliminary evaluation index system: through the analysis of relevant literature and the interpretation of relevant national documents, based on the talent training goals of vocational education and the characteristics and structural elements of vocational education teachers' professional quality, combined with the feedback from expert interviews, using the factor analysis method to determine the indicators and their levels in the professional quality evaluation index system of vocational education teachers and thus obtain the preliminary evaluation index system, as shown in Table 1.

## 4. Experiment and Analysis

### 4.1. Data Samples and Preprocessing

In order to experimentally verify the model proposed in this article, a dataset is constructed according to the teacher education evaluation indicators proposed in Chapter 3, which includes 1600 sets of data. In order to process the data more conveniently and quickly, and at the same time, in order to reduce the adverse impact on the model due to the difference in dimensions between the data and consider its impact on the actual evaluation value, we change the dimensional data into infinite. The data of the class is mapped, and the data is mapped to the range of 0 to 1 for processing, and the samples are normalized. The following is the normalization formula:

(16) $$\begin{array}{c} Y=\frac{X-X_{\min}}{X_{\max}-X_{\min}}. \end{array}$$

### 4.2. Performance Comparison of Improved Algorithms

In order to prove the superiority of the IGWO-BP algorithm proposed in this article, experiments are carried out on IGWO and standard GWO, and the convergence comparison is shown in Figure 3.

As can be seen from Figure 3, the convergence of the IGWO algorithm in the 50th generation is less than 0.005, while the standard GWO algorithm only converges to 0.01 in the 300th generation. It can be seen that the accuracy of the IGWO algorithm has been improved, and the convergence speed is faster than the unimproved GWO algorithm.

After the data in the dataset is normalized to [0, 1], the samples are divided into three categories using a self-organizing mapping algorithm. The training samples, test samples, and test samples account for 60%, 20%, and 20% of the total samples, respectively. The function of the training sample is to train the entire neural network model, the function of the test sample is to prevent “overfitting,” and the function of the test sample is to test the generalization ability of the prediction model.  Figure 4 is a graph showing the fitness comparison between the IGWO-BP model and the GWO-BP model.

It can be seen from Figure 4 that when the IGWO-BP model is iterated to the 20th generation, the mean square error has dropped significantly. When the unoptimized GWO-BP model iterated to the 280th generation, it began to show a more significant decline. Finally, IGWO-BP reaches a lower MSE value earlier than unimproved GWO-BP, which indicates that IGWO-BP converges faster and achieves higher accuracy.

### 4.3. Model Parameter Selection

(1) The influence of the number of samples on network training: in the case of using the same number of hidden layer units and training algorithm, in the same training environment, the number of samples participating in training is set to 500 and 1000, respectively. Train the neural network with an existing dataset and observe the effect of the variable on the network. Perform simulation training in the neural network toolbox, observe the training results, and draw the training process as shown in Figure 5.

As can be seen from the figure, as the number of training samples increases, the gap between the training set, the validation set, and the test set becomes smaller and smaller. When the number of samples is 500, it can be clearly observed that the gap between the training set, the test set, and the validation set is relatively large. When the number of training samples is expanded to 1000, when the training has progressed to a certain extent and is about to end, the training set and the validation set basically overlap, indicating that there is not much error in the number of samples in the two groups during training. This situation shows that when there are too few training samples, the gap between the accuracy on the training set and the MSE on the test set and validation set is too large, and it is difficult to use the neural network trained on the training set to diagnose the samples on the validation set and the test set.

(2) In the case of using the same number of samples and training algorithm, in the same training environment, the number of neurons in the hidden layer participating in the training is set to 5–15, respectively. The training results obtained are shown in Figure 6. It can be seen that when the number of neurons in the hidden layer is 12, the MSE is the smallest, so the number of hidden layers is selected as 12.

### 4.4. Model Performance Verification

The data from the test set was fed into the IGO-BP model to demonstrate its efficacy in assessing the professional quality of teacher education.  Table 2 shows the comparison of the acquired findings with the expert assessment results. This article's output findings are quite near to the expert assessment results, and the error is very minimal. Consequently, this article's suggested model for measuring the professional quality of teacher education performs high accuracy.

### 4.5. Influence of TES Integrating PMH on Teachers' Professional Quality

In order to prove the superiority of the diversified and open TES management system that integrates public mental health proposed in this paper, this article selects three evaluation indicators of professional quality of teacher education to compare the changes before and after the integration of public mental health. The results obtained are shown in Figure 7. The results show that the proposed multidimensional and open TES management system integrating public mental health can effectively improve the professional quality of teachers in all aspects.

## 5. Conclusion

The teacher education management system is crucial to the operation of the TES. It is the core institutional system of the TES, which stipulates the management authority and functional scope of the relevant departments of the TES. After the new pluralistic and open TES is formed, the original management system must be adjusted accordingly. Straighten out the relationship between various interest departments, divide the management authority of each management department, clarify their respective functional scope, clarify their respective rights and responsibilities, and standardize the behavior of management departments. In order to perform their duties, maintain and promote the virtuous circle of teacher education, ensure the healthy, orderly, and high-quality development of teacher education, and improve the efficiency of teacher education. If the management system is not adjusted in time and the relationship between various interest departments is not well coordinated, it will inevitably lead to confusion in the management of teacher education, unclear functions, and prevarication, and thus affect the work efficiency and training quality of teacher education. The public psychology course for normal students has a clear mission of serving teacher education. Teachers should always grasp this basic teaching direction in the design of practical teaching and focus on the characteristics of teacher education. In teaching, the focus should be on helping normal students learn psychology from practical teaching situations, improving their ability to use psychological thinking to think and understand educational and teaching problems and to use psychological knowledge and principles to solve practical educational and teaching problems. In this context, this article integrates public mental health (PMH) into the diversified and open management system of TES, then uses a neural network to evaluate and complete the following tasks: (1) this article introduces the development status of diversified and open TES management systems at home and abroad and the importance of public psychology courses to teacher education. (2) The framework of TES integrating PMH is proposed, and then the principles of BPNN and gray wolf optimization (GWO) algorithm are introduced, and the IGWO-BPNN model is constructed accordingly. (3) The convergence and fitness of the IGWO-BP model and the GWO-BP model are compared through experiments, which proves the superiority of the performance of the IGWO-BP model. The optimal model is constructed by selecting parameters, and then the output of the model is compared with the expert evaluation results, and the error is small. It is proved that the model has superior performance in evaluating the professional quality of teacher education. (4) This article selects three professional quality evaluation indicators of teacher education to compare the changes before and after the integration of PMH. The results show that the proposed diversified and open management system of TES integrating PMH can effectively improve the professional quality of teachers in all aspects.

## Figures and Tables

**Figure 1:** The framework of TES integrating public mental health.

**Figure 2:** The basic structure of the BP neural network.

**Figure 3:** Convergence comparison of IGWO and standard GWO algorithms.

**Figure 4:** The fitness comparison of IGWO-BP and GWO-BP neural network.

**Figure 5:** The effect of the model when the number of training samples is 500 and 1000.

**Figure 6:** Changes in the number of neurons in the hidden layer and MSE.

**Figure 7:** Comparison of evaluation indicators before and after integrating PMH.

**Table 1:** Teacher education evaluation index integrating public mental health.

Index	Label
Teaching with the help of psychology-related video clips	T1
Let students learn by doing experiential classroom mental games	T2
Create psychological situations for specific content for students to practice	T3
Let students use psychology to solve problems according to teaching content	T4
Lectures are interesting	T5
Creative teaching thinking	T6
Dare to challenge challenges and have no regrets about education	T7
Conscientiously complete teaching tasks and actively participate in reforms	T8
Treat students fairly	T9
Strictly require students to teach students in accordance with their aptitude	T10
Master the methods of organizing students to carry out practical training	T11
Guide students to participate in skill competitions and graduation thesis	T12
Using multiple evaluation methods to evaluate student development	T13
Design teaching objectives and plans according to training objectives	T14
Promote the spirit of science and abide by academic norms	T15

**Table 2:** The output of the model is compared with the expert evaluation results.

Number	1	2	3	4	5	6	7	8
IGO-BP output	0.846	0.815	0.752	0.635	0.921	0.688	0.729	0.869
Expert results	0.851	0.814	0.752	0.634	0.919	0.686	0.731	0.870

## Data Availability

The datasets used during the current study are available from the author on reasonable request.
